# Potential drug-drug interactions and associated factors among admitted patients with psychiatric disorders at selected hospitals in Northwest Ethiopia

**DOI:** 10.1186/s40360-022-00630-1

**Published:** 2022-11-30

**Authors:** Ephrem Mebratu Dagnew, Asrat Elias Ergena, Samuel Agegnew Wondm, Ashenafi Kibret Sendekie

**Affiliations:** 1 Depatment of Pharmacy, College of Health Sciences, Debre Markos University, Debre Markos, Ethiopia; 2 Department of Pharmaceutical Chemistry, School of Pharmacy, College of Medicine and Health Sciences, University of Gondar, Gondar, Ethiopia; 3 Depatment of Clinical Pharmacy, School of Pharmacy, College of Medicine and Health Sciences, University of Gondar, Gondar, Ethiopia

**Keywords:** Drug-drug interactions, Psychiatric disorders, Severity, Northwest Ethiopia

## Abstract

**Background:**

Prescribing medications without potential drug-drug interactions (pDDIs) is one of the components of the rational use of medications. However, taking combined medications has resulted in life-threatening pDDIs, which are causing severe clinical outcomes for patients. This study was aimed at assessing the prevalence of pDDIs and associated factors in admitted patients with psychiatric disorders.

**Methods:**

An institution-based multicenter cross-sectional study was conducted among patients with psychiatric disorders admitted to a selected hospital in Northwest Ethiopia. Samples were approached through a systematic sampling method. The Statistical Package for the Social Sciences (SPSS) version 26 was used to analyze the data. Logistic regression was applied to determine the association of variables with pDDIs. A *p*-value of < 0.05 was statistically significant.

**Results:**

Out of 325 study participants, more than half (52.9%) were females, with a median age of 61 years. Overall, more than two-thirds (68.9%) were exposed to at least one clinically significant, either significant or serious level of pDDIs. Nearly one-fourth (23.2%) of participants had at least one serious level of pDDIs. Older patients were found more likely to have pDDIs compared to younger patients (*p* = 0.043). Similarly, patients with a higher number of prescribed medications (*p* = 0.035) and patients with longer hospital admissions (*p* = 0.004) were found more likely to be exposed to pDDIs than their counterparts.

**Conclusion:**

In this study, a significant number of admitted patients with psychiatric problems encountered clinically significant pDDIs. As a result, healthcare providers could assess and follow patients with a combination of medications that potentially have a drug-drug interaction outcome.

## Introduction

Medications have a potential contribution to negative treatment outcomes unless appropriately used. Thus, the morbidity and mortality of patients with a series of medical illnesses has been significantly affected by inappropriate medication use [1]. Drug-drug interaction, among different medication-related problems, can occur when the effect of one drug is altered by another drug, including a concomitant treatment, over-the-counter medication, food, or substance, like alcohol or tobacco [2]. As a result, a drug-drug interaction can be defined as the pharmacological response to the administration or co-exposure of one drug with another drug that modifies the response of patients to the drug effect [3]. The consequences of clinically significant pDDIs have a negative impact on the morbidity, mortality, duration of hospitalization, quality of life, and healthcare costs of the patients [4].

A clinically relevant drug-drug interaction occurs when the effectiveness or toxicity of one medication is altered by the administration of another medication or a substance that is administered for medical purposes (to be distinguished from drug-food interactions). Adverse consequences of drug-drug interactions may result from either diminished therapeutic effect or toxicity [5]. Drug-drug interactions (DDIs) are becoming an increasingly important cause of adverse drug reactions. It has been reported that 20 − 30% of all adverse reactions to drugs are caused by drug-drug interactions, which can be prevented through appropriate monitoring and follow-up. But this incidence increases among the elderly and patients who take two or more medications [2].

Drugs for psychiatric disorders that result in serum concentration changes are generally most relevant for drugs with a narrow therapeutic index. These drugs include lithium and clozapine, where increases or decreases play a role in worsening clinical conditions or increasing the risk of serious adverse effects [6].

The most serious interactions with psychotropics result in profound sedation, central nervous system toxicity, large changes in blood pressure, ventricular arrhythmias, and an increased risk of dangerous side-effects or a decreased therapeutic effect of one of the interacting drugs [7, 8]. It is difficult to completely prevent drug-drug interactions, especially in patients with psychiatric problems, due to the lifelong treatment use of multidrug regimens and the fact that most patients are elderly. Close monitoring of highly at-risk patients may prevent life-threatening outcomes. Nowadays, drug-drug interactions are among the major challenges in patients with psychiatric disorders. Monitoring and reporting of these DDIs in medications used for psychiatric problems is necessary due to the pharmacokinetic and pharmacodynamic nature of the drugs. However, in Ethiopia, the investigations regarding the prevalence and nature of pDDIs in admitted patients with psychiatric disorders are limited. Even though there is a single study that demonstrated drug-drug interactions in patients with psychiatric disorders, it was a single-center study with a retrospective cross-sectional design [8]. The current multicenter study was part of a project initially published regarding the prevalence of drug-related problems (DRPs) [9]. The initial study couldn’t address a detailed investigation of the extent of drug-drug interactions and its determinants. Therefore, this study assessed the prevalence of potential drug-drug interactions and associated factors among admitted patients with psychiatric disorders in selected hospitals in Northwest Ethiopia. The study also analyzed the severity of existing drug-drug interactions.

## Methods

### Study design and setting

An institutional-based multicenter cross-sectional study was conducted from April to July 2021 at five comprehensive and specialized hospitals in Northwest Ethiopia. These hospitals include the University of Gondar Comprehensive and Specialized Hospital (UoGCSH), Felege-Hiwot Comprehensive and Specialized Hospital (FHCSH), Tibebe-Ghion Comprehensive and Specialized Hospital (TGCSH), Debre-Markos Comprehensive and Specialized Hospital (DMCSH), and Debre-Tabor Comprehensive and Specialized Hospital (DTCSH). These hospitals have provided healthcare services for over 26.5 million people in their total catchment areas.

### Study participants and inclusion criteria

All adult patients with a psychiatric problem who were admitted to the psychiatric wards of selected hospitals in Northwest Ethiopia were included in the study population. Patients aged 18 years or older, diagnosed with any psychiatric disorder and received a combination of medications were included in the study. Pregnant and lactating mothers, critically ill patients who couldn’t respond to self-response interview questions, and patients with incomplete medical records during the study period did not participate in this study.

### Sample size determination and sampling techniques

The single population proportion formula was used to calculate the required sample size by considering the following assumptions: the proportion of drug–drug interactions to be 81.8% (*P* = 0.82) [8], the reliability coefficient for 95% confidence level (Z = 1.96) and 5% margin of error (d = 0.05); *n* = z^2^pq/d^2^.

After adding a 10% contingency of non-response, the total sample size of participants to be selected was 325. Participants from the selected hospitals were included based on a proportional allocation formula: ni = n*Ni/N, where, ni = sample size from each hospital, *n* = total sample size to be selected, *N* = total population, Ni = total population from each selected hospital. Consequently, the total population from all selected study areas was 984 per year (264 from UoGCSH, 192 from FHCSH, 180 from TGCSH, 192 from DMCSH, and 156 from DTCSH) based on the previous admission. Considering this, 87, 63, 60, 63, and 52 study participants were included from the respective hospitals in the final study.

The participants were included in the final study using a consecutive sampling technique, and all eligible participants from respective sites were enrolled consecutively until the required sample size was obtained.

### Definition of terms

Psychiatric disorders: according to the DSM-5 definition, “a syndrome characterized by clinically significant disturbance in an individual’s cognition, emotion regulation, or behavior reflecting a dysfunction in the psychological, biological, or developmental processes underlying mental function.”[10].

Drug-drug interactions: defined as the pharmacological or clinical response to the administration or co-exposure of a drug with another drug that modifies the patient’s response to the drug index [3].

Potential drug-drug interactions: According to Consensus recommendations for systematic evaluation of drug-drug interaction evidence for clinical decision support “a potential DDI is defined as the co-prescription of two drugs known to interact, and therefore a DDI could occur in the exposed patient” [11].

The severity of drug-drug interactions: it is the level of evidence of the severity of the outcome from interactive medications. It can either be contraindicated, the drug-pair is contraindicated in the patient for current use, serious; such an interaction may have a risk of death and/or may result in some serious negative outcome, and recommended to use an alternative, significant; it may have a harmful effect on the patient’s condition and can require close monitoring, or minor (no change required); it may have an increase in frequency or severity of side effects, but would not require therapeutic change and, they are self-limited effects on patients [12].

Comorbidity: is the presence of one or more additional conditions, often co-occurring with the primary condition.

Duration of treatment: refers to how long (in years) a patient was treated with a manual method for any given problem.

### Data collection instruments, procedures and quality management

The data was collected using a structured English questionnaire developed after reviewing various literature [13–21]. It was collected by both patient interviews and retrospective medical recording methods for primary and secondary data, respectively. Patient socio-demographic characteristics include: age, gender, monthly income, alcohol drinking habit, substance use (Khat and cigarettes), educational level, occupations, residency, etc. Whereas medications and clinical characteristics like history of allergy, type of medication, number of medications, the duration of treatment, presence of comorbidities, type of psychiatric disorders, and number of hospitalizations were also extracted from the medical records of the participants. Data were collected by five trained clinical pharmacists and five trained psychiatric nurses, who were overseen by two clinical pharmacy lecturers. The chart numbers were entered into Microsoft Office Excel 2016 and checked for duplication.

To ensure the quality of the data, data collectors were trained for two days, and orientation was also provided by the principal investigator. The principal investigator (PI) closely supervised the data collection process, and the collected data was checked daily for completeness during the data collection period. The data collection tool was pretested on 5% of the calculated sample size of patients admitted to the psychiatric ward of Dessie comprehensive specialized hospital to check the acceptability and consistency of the data collection tool two weeks before the actual data collection. The data from the pretest was excluded in the analysis. The questionnaire was sent to senior clinical pharmacists and senior physicians, who were academicians and researchers, for face validity and approval.

### Data entry and statistical analysis

The data was coded, cleared, and checked for completeness before being entered into EPI-data version 4.6 and exported to the statistical software package for social sciences (SPSS) version 26 for analysis. Then, it was reviewed and cleaned manually for its completeness and consistency. The results were summarized using descriptive statistics including frequency and percentage for categorical and mean and standard division for continuous variables. The Medscape drug-interaction checker was used to check for pDDIs. To make the assessment of the existing pDDIs consistent, the severity of identified drug-drug interactions was also characterized using evidence from Medscape. Finally, we analyzed only clinically significant drug-drug interactions with most of the pDDIs resulting in significant and serious levels of drug-drug interactions. Independent variables having a *p*-value < 0.25 in the univariate logistic regression analysis entered into the multivariable logistic regression analysis to control the confounding effect. The odds ratio (OR) with a 95% confidence interval was also computed. In the final model, a *p*-value < 0.05 was statistically significant.

## Results

### Socio-demographic characteristics of the study participants

More than half (172, or 52.9%) of the study participants were females, with a median age of 61 (24–85) years. The majority of the participants were rural residents; 215(66.2%). More than half, 173 (53.2%), of the participants had no regular monthly income and the majority of the respondents were substance non-users, 319 (98.2%) (Table 1).

**Table 1:** Socio-demographic characteristics among patients with psychiatric disorders admitted in selected hospitals of Northwest Ethiopia from April –July, 2021 (*N* = 325)

Variables	Category	Frequency (%)	Median (range)
Sex	Male	153(47.1)	
	Female	172(52.9)	
Age in years	18–30	89(27.4)	61(24–85)
	31–45	115(35.4)	
	46–60	71(21.8)	
	≥ 61	50(15.4)	
Residency	Rural	215(66.2)	
	Urban	110(33.8)	
Educational status	Non-formal education	108(33.2)	
	Primary education	106(32.6)	
	Secondary	61(18.8)	
	College and university	50(15.4)	
Monthly income (Eth birr)	< 1500	27(8.3)	
	1500–2499	38(11.7)	
	2500–3499	35(10.8)	
	≥ 3500	52(16)	
	No regular income	173(53.2)	
Substance use (Khat, cigarette)	Yes	6(1.8)	
	No	319(98.2)	
Alcohol drinking habit	Yes	33(10.2)	
	No	292(89.8)	

### Clinical characteristics of the study participants

Regarding the types of psychiatric disorders, schizophrenia 140 (30.8%) was responsible for the admission of a greater proportion of patients. More than half of the participants, 182 (56%), had comorbid conditions in addition to psychiatric disorders. The majority of the study participants, 290 (89.2%), were admitted for more than a week. The study participants received an average of 3 (ranges 1–8) medications per patient (Table 2).

**Table 2:** Clinical characteristics of the study participants

Variables	Category	Frequency, n (%)	Median (range)
Types of psychiatric disorders at admission	Schizophrenia	140(30.8)	
	Brief-psychotic feature	117(25.7)	
	Bipolar disorder	67(14.7)	
	Major mood disorder	55(12.1)	
	Other^a^	8(2.5)	
Presence of comorbidities	No	143(44)	
	Yes	182(56)	
Types of comorbidities	Heart failure	6(1.8)	
	Substance use	6(1.6)	
	Peptic ulcer disease	5(1.5)	
	Retroviral infection (HIV)	3(0.9)	
	Tuberculosis (TB)	2(0.6)	
Hospital stays (days)	< 7	35(10.8)	14(3–35)
	≥ 7	290(89.2)	
Number of prescribed medications	< 5	184(56.6)	3 (1–8)
	≥ 5	141(43.4)	
Duration of treatment	≤ 1 year	176 (54.1)	
	2–3 years	86 (26.5)	
	≥ 4 years	63 (19.4)	

Others^a^, substance-related disorders, anxiety disorders, post-traumatic disorders

### Prevalence of potential drug-drug interaction and distribution based on severity

A higher proportion of study participants (107, 33%) had 1 to 3 pDDIs. This study showed that the overall prevalence of the pDDIs was found to be 68.9%, which revealed that a total of 224 participants were encountered with at least one serious or significant pDDIs, with a median (range) of 3 (1–7) pDDIs per patient. Regarding the severity of pDDIs near one-fourth, 52 (23.2%) of the participants had serious drug-drug interactions (Table 3).

**Table 3:** Prevalence and severity of potential drug-drug interactions among the study participants

Variables	Category	Frequency, n (%)	Median (range)
Prevalence of pDDIs	1–3	107(33%)	3 (1–7)
	4–5	84(25.8%)	
	≥ 6	33(10.2%)	
	Total	224 (68.9%)	
Level (severity) of pDDIs	Serious	52(23.2%)	
	Significant	172(76.8%)	

### Common interacting medications, their level of interaction and adverse outcomes

Patients on a combination of fluoxetine and amitriptyline accounted for a higher proportion of serious pDDIs, 10(4.5%), while a combination of chlorpromazine and trihexyphenidyl was responsible for a higher proportion of patients, 45(20.1%) exposed to significant pDDIs (Table 4).

**Table 4:** Level of pDDIs and potential adverse outcome with respective combined prescribed medications (*N* = 224)

Paired medications	Frequency (%)	Leve of interaction	Adverse outcome
Fluoxetine -Amitriptyline	10(4.5)	Serious	Fluoxetine increases the effect of amitriptyline by affecting CYP2C19. Fluoxetine and amitriptyline both increase serotonin levels. Avoid use in combination.
Carbamazepine-diazepam	8(3.6)	Serious	Carbamazepine will decrease the level or effect of diazepam by affecting hepatic/intestinal enzyme CYP3A4 metabolism. Avoid or Use Alternate Drug.
Carbamazepine-haloperidol	7(3.1)	Serious	Carbamazepine will decrease the level or effect of haloperidol by affecting hepatic/intestinal enzyme CYP3A4 metabolism. Avoid or Use Alternate Drug.
Fluoxetine-Risperidone	6(2.7)	Serious	Fluoxetine will increase the level or effect of risperidone by affecting hepatic enzyme CYP2D6 metabolism. Avoid or Use Alternate Drug.
Fluoxetine-Haloperidol	5(2.2)	Serious	Fluoxetine will increase the level or effect of haloperidol by affecting hepatic enzyme CYP2D6 metabolism. Avoid or Use Alternate Drug.
Chlorpromazine-Amitriptyline	5(2.2)	Serious	Chlorpromazine and amitriptyline both increase QTc interval. Avoid or Use Alternate Drug.
Chlorpromazine-Haloperidol	4(1.8)	Serious	chlorpromazine and haloperidol both increase QTc interval. Avoid or Use Alternate Drug.
Fluoxetine-cimetidine	4(1.8)	Serious	Fluoxetine will increase the level or effect of cimetidine by affecting hepatic enzyme CYP2C19 metabolism. Avoid or Use Alternate Drug.
Fluphenazine deaconate-haloperidol	3(1.3)	Serious	fluphenazine and haloperidol both increase QTc interval. Avoid or Use Alternate Drug.
Chlorpromazine-Trihexyphenidyl	45(20.1)	Significant	Chlorpromazine increases effects of trihexyphenidyl by pharmacodynamic synergism. Use Caution/Monitor. Potential for additive anticholinergic effects.
Haloperidol-Trihexyphenidyl	32(14.3)	Significant	haloperidol increases effects of trihexyphenidyl by pharmacodynamic synergism. Use Caution/Monitor. Potential for additive anticholinergic effects.
Trifluoperazine-trihexyphenidyl	25(11.2)	Significant	trifluoperazine increases effects of trihexyphenidyl by pharmacodynamic synergism. Use Caution/Monitor. Potential for additive anticholinergic effects.
Fluphenazine decanoate-trihexyphenidyl	22(9.8)	Significant	Fluphenazine increases effects of trihexyphenidyl by pharmacodynamic synergism. Use Caution/Monitor. Potential for additive anticholinergic effects.
Fluoxetine- Amitriptyline	10(4.5)		Amitriptyline and fluoxetine both increase QTc interval. Modify Therapy/Monitor Closely.
Carbamazepine-diazepam	8(3.6)	Significant	Carbamazepine decreases levels of diazepam by increasing metabolism. Use Caution/Monitor.
Carbamazepine-haloperidol	7 (3.6)	Significant	Carbamazepine decreases levels of haloperidol by increasing metabolism. Use Caution/Monitor.
Fluoxetine-Risperidone	6(2.7)	Significant	Fluoxetine and risperidone both increase QTc interval. Use Caution/Monitor.
Fluoxetine-Haloperidol	5(2.2)	Significant	Fluoxetine and haloperidol both increase QTc interval. Modify Therapy/Monitor Closely.
Chlorpromazine-Amitriptyline	5(2.2)	Significant	Chlorpromazine and amitriptyline both increase sedation. Use Caution/Monitor.
Chlorpromazine-Haloperidol	4(1.8)	Significant	-Chlorpromazine and haloperidol both increase sedation. Use Caution/Monitor. -chlorpromazine and haloperidol both increase antidopaminergic effects, including extrapyramidal symptoms and neuroleptic malignant syndrome. Use Caution/Monitor.
Fluphenazine-haloperidol	3(1.3))	Significant	Fluphenazine and haloperidol both increase sedation. Use Caution/Monitor. -Fluphenazine and haloperidol both increase antidopaminergic effects, including extrapyramidal symptoms and neuroleptic malignant syndrome. Use Caution/Monitor.

### Factors associated with the occurrence of potential drug-drug interactions

Logistic regression analysis was performed to examine the relationship between existing pDDIs and the number of predictor variables. Multivariable logistic regression revealed that age, number of drugs, and hospital stay were independently associated with the occurrence of pDDIs in admitted patients with psychiatric disorders. Consequently, it has been found that, holding all other predictor variables constant, the odds of pDDIs in elderly patients with an age greater than or equal to 61 is about 1.5 times [AOR = 1.47, 95% CI (1.13–2.56); *p* = 0.043] compared with patients aged 18–30 years old. Similarly, patients with a higher number of prescribed medications and those who stayed longer at the hospital were found more likely to be exposed to pDDIs than their counterparts, [AOR = 2.75, 95% CI (1.56–7.31); *p* = 0.035] and [AOR = 2.13, 95% CI (1.34–3.64); *p* = 0.004], respectively (Table 5).

**Table 5:** Univariable and multivariable analyzes of factors associated with pDDIs

Variables	Category	Potential Drug-drug interaction		COR (95% CI)	AOR (95% CI)	*P*-value
		No	Yes			
Age (Years)	18–30	22	67	1	1	
	31–45	43	72	0.55(0.13–1.89)	0.39(0.17–2.65)	
	46–60	27	44	0.54(0.09–1.02)	0.36(0.12–1.86)	
	≥ 61	9	41	1.5(1.01–2.65)	1.47(1.13–2.56)	0.043*
Sex	Male	49	104	1	1	
	Female	52	120	0.92(0.24–2.16)	1.48(0.96–2.28)	0.62
Source of medication	Free Payment	61 40	134 90	1 0.98(0.17–2.04)	1 1.24(0.72–2.11)	0.429
Presence of Comorbidities	No	36	107	1	1	
	1–2	21	47	1.33(0.76–2.25)	1.74(0.90–3.36)	0.098
	3–4	32	61	1.56(0.28–4.74)	1.12(0.74–2.47)	0.076
	≥ 5	12	9	3.96(0.32–18.45)	1.16(0.98–2.13)	0.087
Number of prescribed medications	< 5 ≥ 5	56 45	128 96	1 1.07(1.002–1.761)	1 2.75(1.56–7.31)	0.035*
Duration of treatment	≤ 1 year 2–3 years ≥ 4 years	56 25 20	120 61 43	1 0.88(0.15–2.67) 0.99(0.25–2.61)	1 0.67(0.35–1.40) 0.83(0.35–1.78)	0.31 0.57
Length of hospital stay	< 7days ≥ 7 days	85 16	205 19	1 2.03(0.56–3.12)	1 2.13(1.34–3.64)	0.004*

*COR* Crude odds ratio, *AOR* Adjusted odds ratio

*denotes statistically significant at *p* < 0.05

## Discussion

Prescribing medications without potential drug-drug interactions is a component of the rational use of medications. Drug-drug interactions continue to be a major cause of morbidity and mortality of admitted patients [22]. Administration of more than or equal to two drugs for an admitted patient repeatedly leads to pDDIs, which may further compromise the patient’s health-related outcome. To the best of the authors’ literature search, the prevalence and extent of potential drug-drug interactions in admitted patients with psychiatric disorders have not been investigated in the study areas. Therefore, this facility-based multicenter study was conducted to determine the prevalence of potential drug-drug interactions and the severity of the existing drug-drug interactions using the Medscape drug-drug interaction checker in admitted patients with psychiatric disorders.

Overall, nearly two-thirds (68.9%) of the study participants had clinically significant pDDIs, which is consistent with the previous studies [21, 23, 24]. The finding suggests that a higher proportion of patients have at least one significant potential drug-drug interaction. Therefore, patients taking a combination of potentially interactive medications need close follow-up. In contrast, the current finding is lower than studies demonstrated in Mekelle, Ethiopia [8]. The discrepancy in the prevalence of pDDIs among different studies might be related to differences in healthcare approach with pharmacist involvement, differences in alternative medication availability, and differences in the use of software or tools to identify pDDIs in these patients taking interactive medications. Additionally, the current study is a multicenter study that may differ from a single study due to differences in pharmaceutical care across the settings.

Based on the severity of consequence outcomes resulting from interactive medications, the level of pDDIs is commonly classified as contraindicated, major, significant, and minor. In this study, we analyzed potential drug-drug interactions, which were relevant in terms of clinical outcome and quality of life of the patients. Consistent with the previous studies [8, 21, 23, 24], most study participants were exposed to clinically significant pDDIs, either with serious or significant drug-drug interactions, which needed interventions. Interactive medications may be prescribed because of the non-availability of alternative medications with less interaction potential or due to the knowledge and skill gap of healthcare practitioners about the pharmacokinetics and dynamics properties of the medications. Therefore, healthcare providers, particularly prescribers, could be vigilant about the combination of medications, which can lead to life-threatening treatment and clinically significant interactions. The use of alternative medications with a low potential for interaction could be recommended. Close monitoring and follow-up of patients who received interactive medication is also strongly advised.

The occurrence of drug-drug interactions may have many contributing factors. The current findings from multivariate logistic regression revealed that being elderly, being treated with a higher number of drugs, and longer hospital stays were significantly associated with the presence of pDDIs. In line with the previous studies [24, 25], compared with younger patients (18–30 years), older patients with an age greater than or equal to 61 years were found more likely to be exposed to pDDIs. This finding might be justified by the fact that patients of advanced age may have multimorbidity and comorbidities with polypharmacy, which can be responsible for potential drug-drug interactions. Age-related changes in pharmacokinetic properties of the drug may also be responsible for pDDIs. The elderly psychiatric population is particularly prone to being on many drugs, including psychotropic, which increases the potential for a harmful drug-drug interaction [25]. These findings suggest that elderly patients need to be under close monitoring and follow-up with healthcare providers.

In line with the previous studies [2, 21, 24], the current finding also revealed that patients treated with a higher number of medications were more likely to be exposed to pDDIs. As a result, patients with a higher number of medications could be assessed accordingly, and healthcare providers could be highly vigilant in the prevention of harmful drug-drug interactions with patients taking a higher number of medications with potentially interactive combinations. Patients with longer hospital stays were also found more likely to have a higher incidence of pDDIs compared with patients with shorter hospital stays. This is consistent with the previous studies [21]. Patients admitted to different levels of hospitals may be exposed to different medications, and patients with a longer hospital stay may be repeatedly exposed to different medications, which may result in a drug-drug interaction. This finding suggests that patients with a longer hospital stay could be assessed for the potential medication interactions and pharmacists would be better involved to intervene and tailor recommendations based on the available medications with a low potential interaction.

Generally, the current study has highlighted the level of pDDIs and potential associated factors among patients with psychiatric disorders, which can be a benchmark for future investigators with prospective studies in larger populations. Drug-drug interactions may not be avoidable, but the existing life-threatening pDDIs may be minimized through close monitoring and follow-up of risky patients. The prevention of pDDIs and achieving good treatment outcomes for non-significant and preventable DDIs needs multifactorial involvement, including healthcare providers and patients, starting with the prescribing and use of prescribed medications, availing of alternative medications with less interaction potential, and assessing the significance of interactive medications using interaction checker software and tools. Documentation of the existing pDDIs could also be improved. Therefore, assessing and following patients with a combination of medications which potentially have a drug-drug interaction could be a must to achieve a better treatment outcome.

The current study has some limitations. The first thing is that since the study is cross-sectional, it couldn’t show a real cause-outcome association and it did not analyze the consequences of the pDDIs. The second thing is that the results may not be used to generalize for the entire country. However, it may be used as a benchmark for future studies in the country. Therefore, prospective studies in a larger sample population could be recommended.

## Conclusion

The current study highlighted that a significant number of admitted patients with psychiatric disorders were exposed to clinically significant pDDIs. Older patients, patients with a higher number of medications, and patients with a longer hospital stay were more likely to have pDDIs compared with their counterparts. Therefore, healthcare providers could assess and follow patients with such risk factors with a combination of medications that potentially have a drug-drug interaction outcome. Minimize the occurrence of life-threatening and clinically significant pDDIs by using rational medication prescription and patient monitoring could be a role for healthcare providers.

## Data Availability

The datasets generated and/or analyzed during the current study are not publicly available to protect from unnecessary abuse of full data of the participants but are available from the corresponding author on reasonable request.

## Abbreviations

DDI: Drug-drug interactions
pDDIs: potential drug-drug interactions
